# Atractylenolide III Attenuates Apoptosis in H9c2 Cells by Inhibiting Endoplasmic Reticulum Stress through the GRP78/PERK/CHOP Signaling Pathway

**DOI:** 10.1155/2022/1149231

**Published:** 2022-09-14

**Authors:** Meng-yu Zuo, Tong-juan Tang, Xiang Wang, Jin-fan Gu, Liang Wang, Jian Chen, Juan Yao, Xiang-yang Li, Peng Zhou, Jin-ling Huang

**Affiliations:** ^1^School of Traditional Chinese Medicine, Anhui University of Chinese Medicine, Hefei 230012, Anhui, China; ^2^Department of Integrated Traditional Chinese and Western Medicine, Anhui University of Chinese Medicine, Hefei 230012, Anhui, China; ^3^Research Institute of Integrated Traditional Chinese and Western Medicine, Anhui Academy of Chinese Medicine, Hefei 230012, Anhui, China

## Abstract

The objective of this study was to determine the effect of atractylenolide III (ATL-III) on endoplasmic reticulum stress (ERS) injury, H9c2 cardiomyocyte apoptosis induced by tunicamycin (TM), and the GRP78/PERK/CHOP signaling pathway. Molecular docking was applied to predict the binding affinity of ATL-III to the key proteins GRP78, PERK, IRE*α*, and ATF6 in ERS. Then, in vitro experiments were used to verify the molecular docking results. ERS injury model of H9c2 cells was established by TM. Cell viability was detected by MTT assay, and apoptosis was detected by Hoechst/PI double staining and flow cytometry. Protein expression levels of GRP78, PERK, eIF2*α*, ATF4, CHOP, Bax, Bcl-2, and Caspase-3 were detected by Western blot. And mRNA levels of GRP78, CHOP, PERK, eIF2*α*, and ATF4 were detected by RT-qPCR. Moreover, the mechanism was further studied by using GRP78 inhibitor (4-phenylbutyric acid, 4-PBA), and PERK inhibitor (GSK2656157). The results showed that ATL-III had a good binding affinity with GRP78, and the best binding affinity was with PERK. ATL-III increased the viability of H9c2 cells, decreased the apoptosis rate, downregulated Bax and Caspase-3, and increased Bcl-2 compared with the model group. Moreover, ATL-III downregulated the protein and mRNA levels of GRP78, CHOP, PERK, eIF2*α*, and ATF4, consistent with the inhibition of 4-PBA. ATL-III also decreased the expression levels of PERK, eIF2*α*, ATF4, CHOP, Bax, and Caspase-3, while increasing the expression of Bcl-2, which is consistent with GSK2656157. Taken together, ATL-III could inhibit TM-induced ERS injury and H9c2 cardiomyocyte apoptosis by regulating the GRP78/PERK/CHOP signaling pathway and has myocardial protection.

## 1. Introduction

Heart failure (HF) is the end-stage manifestation of different types of cardiovascular disease, due to disorders of the systolic function and/or diastolic function of the heart, which affects about 38 million people worldwide and is the leading cause of mortality globally [1]. Endoplasmic reticulum stress (ERS)-induced cardiomyocyte apoptosis exists in the pathological process of HF, which is one of the pathogenesis of HF [2]. Despite advances in current drugs for the treatment of HF, the prognosis remains dismal, and patients treated according to current guidelines are at a higher risk of survival. Therefore, the development of new targeted therapies and the selection of appropriate therapeutic interventions are of great importance for the treatment of HF.

HF has been causally associated with disruption of endoplasmic reticulum (ER) depletion. ERS has recently emerged as a key etiology of cardiovascular disorders, including heart failure [1]. ER is a multifunctional organelle that plays a critical role in lipid, carbohydrate, and protein modification and synthesis, as well as determining cell survival and death [3]. It also plays a major role in a variety of physiological activities. If ERS is severe or lasts for a long time, cells will die. Recent research has shown that ER-induced apoptosis plays a role in the pathophysiology of HF [4]. The ERS occurs when misfolded proteins accumulate in the cavity of ER, which is called the unfolded protein reaction (UPR) [5]. Moderate UPR can reduce the cell injury caused by ERS, but continuous and excessive ERS can cause severe cell damage that is difficult to recover from, promoting the apoptotic mechanism and causing a variety of pathological events [6]. Glucose-regulated protein 78 (GRP78), the ER molecular partner, dissociates from the three ER transmembrane sensors, inositol requiring kinase 1 (IRE1), activating transcription factor 6 (ATF6), and protein kinase-like ER kinase (PERK), triggering the apoptotic cascade. Loss of ER homeostasis is the pathological basis of cardiovascular diseases. Persistent and severe ERS induces myocardial cell apoptosis, which is one mechanism responsible for the pathogenesis of HF [7, 8]. As a result, suppression of ERS could be a major concern for HF [9].

Traditional Chinese medicine (TCM) has multicomponents and multitargets to regulate the body as a whole, which has advantages in reducing adverse effects and improving patients' quality of life, and has been reported to be effective in treating HF [10]. Ling-Gui-Zhu-Gan decoction (LGZGD) is an effective treatment prescribed for HF [11], which is a common Chinese medicine for treating HF in our previous studies. In vivo and in vitro experiments have found that LGZGD has antioxidant and anti-inflammatory effects [12, 13] and protects H9c2 cardiomyocytes by reducing apoptosis [12]. Atractylenolide III (ATL-III) is the effective ingredient of *Atractylodes macrocephala*, one of the LGZGD constituent herbs, as well as one of the LGZGD effective blood components [14]. Therefore, we continue to explore the main active components of LGZGD to further reveal its pharmacodynamic substance basis. A variety of biological activities of ATL-III have been reported, including anti-inflammatory, antioxidant, and antimyocardial apoptosis [15–20]. There is evidence that excessive oxidative stress can cause ERS [21], ERS plays an important role in HF, and ATL-III has a protective effect against oxidative stress-induced cardiomyocyte injury. We hypothesized that ATL-III could protect cardiomyocytes by inhibiting ERS, and we used molecular docking to predict the target, followed *by in vivo* investigation to confirm our hypothesis. In this study, we used tunicamycin (TM) [22] to induce ERS model and the potential mechanism was further explored by validating the GRP78/PERK/CHOP signaling pathway.

## 2. Materials and Methods

### 2.1. Materials and Reagents

ATL-III was purchased from Chroma Biotechnology (Chengdu, China). 0.25% trypsin and Hoechst33342/PI stain solution were purchased from Biosharp (Anhui, China). Tunicamycin was purchased from ACMEC (Shanghai, China). MTT solution was purchased from Zhenwo (Shanghai, China). AnnexinV-FITC/PI Cell Apoptosis Detection Kit was purchased from Servicebio (Wuhan, China). GRP78 (^#^ABM40216), CHOP (^#^ABP50978), PERK (^#^ABP52177), p-PERK (^#^ABP50528), and eIF2*α* (^#^ABP51245) antibody were purchased from Abbkine (Wuhan, China). ATF4 (^#^DF6008) antibody was purchased from Affinity (CHangzhou, China), and p-eIF2*α* (^#^A13982) antibody was purchased from Alpha Applied Bioscience (Beijing, China). Bcl-2 (^#^ab196495) and Bax (^#^ab189491) polyclonal antibody were purchased from Abcam (Cambridge, UK). Caspase-3 (^#^108132117) antibody was purchased from Wanleibio (Shenyang, China). GAPDH (^#^KK0425) antibody was purchased from ZEN-BIOSCIENCE (Chengdu, China). Goat anti-rabbit IgG (^#^A21020) and Rabbit anti-mouse IgG (^#^A21010) were purchased from Abbkine (Wuhan, China). 4-Phenylbutyric acid (4-PBA) was purchased from G-CLONE (Beijing, China). GSK2656157 was purchased from TOPSCIENCE (Shanghai, China). The penicillin/streptomycin was purchased from Sigma (USA).

### 2.2. Molecular Docking

Autodock 4.1 software was used to predict the binding affinity between ATL-III and ERS-related targets [23]. Since water molecules play a key role in the ligand stability at the reactive site, all water molecules in the structure of the crystal are retained during the docking process; finally, ATL-III was docked into the cavity of the corresponding receptor and the best conformation was selected for the binding mode analysis. According to the binding free energy, ATL-III was clearly bound to the target site, and the docking results were displayed in Pymol.

### 2.3. Cell Culture and Treatment

H9c2 cells were cultured in DMEM with 10% FBS and 100U penicillin/streptomycin at 37°C, 5% CO_2_ incubator. Cells were classified into control group, model group, ATL-III (15 *µ*mol/L) group, ATL-III (30 *µ*mol/L) group, and ATL-III (60 µmol/L) group. ATL-III group was pretreated with different concentrations of ATL-III for 24 h. After pretreatment, cells in the model group and ATL-III group were further treated with TM (2 *μ*mol/L) for 24 h.

To further explore the role of the GRP78/PERK/CHOP signaling pathway in the protective effects of ATL-III against HF, the cells were divided into control group, model group, ATL-III group (pretreatment with 60 *μ*mol/L ATL-III for 24 h), ATL-III+ 4-PBA group (ATL-III was pretreated for 23 h and then 1 *μ*mol/L 4-PBA was added for 1 h), ATL-III + GSK2656157 group (ATL-III was pretreated for 23 h and 10 *μ*mol/L GSK2656157 was added for 1 h), 4-PBA group (after 23 h of DMEM culture, cells were treated with 1 mmol/L 4-PBA was added for 1 h), and GSK2656157 group (after 23 h of DMEM culture, cells were treated with 10 *μ*mol/L GSK2656157 added for 1 h). After drug pretreatment, groups were stimulated with TM for 24 h except for the control group, and related indexes were detected.

### 2.4. MTT Assay

H9c2 cells were injected in 96-well plates after being adjusted to a density of 1 × 10^5^ cells/mL. ATL-III (15, 30, 60, 120, and 240 *µ*mol/L) was applied to cells for 24, 48, and 72 h at varying doses. MTT solution (5 mg/mL) was added to each well for 20 *μ*L and incubated for 4 h. The supernatant was removed, and 150 *μ*L of DMSO was added. The absorbance was measured by ATOM spectrometer (Maroche, Italy) at 490 nm and the cell viability was calculated. All experiments were repeated three times.

### 2.5. Apoptosis by Hoechst33342/PI Double Staining

H9c2 cell density was regulated to 1 × 10^5^ cells/mL and inoculated in 6-well plates. After treatment with ATL-III, cells were fixed with 4% paraformaldehyde for 30 min, Hoechst 33342 was added and incubated in the dark for 5 min, washed with PBS 3 times, then PI was added and incubated for 5 min avoiding light. The experiments were observed and recorded under a DMi8 fluorescence microscope (Leica, Germany), and all experiments were repeated three times.

### 2.6. Apoptosis Detection by Flow Cytometry

Cell density was adjusted to 1 × 10^6^ cells/mL and inoculated in 6-well plates. After treatment with ATL-III, H9c2 cells were digested by trypsin (without EDTA) after washing with PBS 3 times. Cell morphology was observed and digestion was completed; then cells were collected and 5 *μ*L of AnnexinV-FITC was added for 15 min at room temperature, followed by 5 *μ*L of PI for 5 min, and detected by flow cytometer (BDFACSCelesta, USA), and analyzed by FlowJo 7.6. All experiments were repeated three times.

### 2.7. Western Blot

RIPA was used to lyse each group of H9c2 cells, and total protein was extracted and quantified by BCA. After electrophoresis, membrane transfer, and closure, GRP78 (1 : 1000), p-PERK (1 : 1000), PERK (1 : 1000), p-eIF2*α* (1 : 1000), eIF2*α* (1 : 1000), ATF4 (1 : 1000), Bcl-2 (1 : 1000), BAX (1 : 1000), Caspase-3 (1 : 1000), and GAPDH (1 : 5000) primary antibodies were added, respectively, overnight at 4°C, and continue incubation for 2 h with the corresponding secondary antibodies. The imaging results were measured with a chemiluminescence image analyzer (Protein Simple, USA), the grayscale values of each band were analyzed by ImageJ software, and all experiments were repeated three times.

### 2.8. RT-qPCR

RNA was first extracted with Trizol after treatment and then reverse-transcribed to cDNA. The reverse transcription conditions were heating at 65°C for 5 min, cooling at 4°C for 1 min, warm bath at 42°C for 60 min, heating at 70°C for 5 min, cooling at 4°C for 1 min, and one cycle. Then real-time PCR (RT-qPCR) was carried out, PCR reaction conditions were predenaturation at 95°C for 300 s, denaturation at 95°C for 15 s, annealing at 60°C for 1 min, extension at 72°C for 30 s, and 40 cycles. GRP78, CHOP, PERK, eIF2*α*, and ATF4 mRNA levels were normalized to *β*-actin by 2^−ΔΔCt^ method, and all experiments were repeated three times. The primers were seen in Table 1.

### 2.9. Statistical Analysis

All statistical analyses were done by using SPSS 23.0 and GraphPad 6.0 software, with the significance level set at *P* < 0.05. One-way analysis of variance (ANOVA) was used for the comparison of multiple groups.

## 3. Results

### 3.1. Molecular Docking

The molecular docking results were expressed as Vina scores, with a low Vina score representing a high degree of binding affinity. ATL-III has a good binding affinity to GRP78 and the best binding affinity to the PERK (Table 2). These results suggest that ATL-III may act effectively on ERS and its related signaling pathway (Figure 1).

### 3.2. Effect of ATL-III on H9c2 Viability

MTT method was applied to evaluate the efficacy of different doses of ATL-III on H9c2 cells proliferation. H9c2 cells were dealt with different doses of ATL-III (15, 30, 60, 120, and 240 *µ*mol/L) for 24, 48, and 72 h. The apoptosis rate was increased when the concentration of ATL-III was 120 *µ*mol/L or 240 *µ*mol/L, and the apoptosis rate was higher when ATL-III was used for 48 and 72 h (Figure 2(a)). Therefore, the follow-up studies were conducted at concentrations of 15, 30, and 60 mol/L for 24 h. The effect of TM on H9c2 cells could be significantly reversed after the intervention of ATL-III, that is, ATL-III treatment significantly reduced the TM-induced apoptosis rate (Figure 2(b)).

### 3.3. Effects of ATL-III on Apoptosis

The apoptosis of H9c2 cells was detected by flow cytometry, Hoechst/PI double staining, and Western blot. Flow cytometry showed that the model group had a higher apoptosis rate than the control group (*P* < 0.01); while the ATL-III (15, 30, 60 mol/L) group had a lower apoptosis rate than the model group (*P* < 0.01) (Figures 3(a) and 3(b)). Hoechst33342 can penetrate the cell membrane and make the normal nucleus appear light blue and the apoptotic cells appear dark blue. PI can make the nucleus appear red through late apoptosis and the death of cells. The findings revealed that the nuclei of H9c2 cells in the model group were bright blue and PI staining was distinctly red compared to the control group, showing the characteristics of apoptosis. While the fluorescence intensity of ATL-III (15, 30, and 60 *μ*mol/L) groups was significantly reduced, the nuclear staining became lighter, and the red color was significantly reduced compared with the model group (Figure 3(c)). Western blot results (Figures 4(d)–4(g)) showed that the expression levels of Bax and Caspase-3 were more significantly increased in the model group than those in the control group (*P* < 0.01), and these expression levels were reversed by ATL-III (*P* < 0.05, *P* < 0.01). The expression of Bcl-2 was significantly lower than that in the control group (*P* < 0.01) and improved after ATL-III treatment (*P* < 0.05, *P* < 0.01). The effects indicate that ATL-III can prevent TM-induced apoptosis in H9c2 cardiomyocytes.

### 3.4. Effects of ATL-III on GRP78, CHOP Protein, and mRNA Expression

Western blot results demonstrated that the protein expression levels of GRP78 and CHOP were significantly higher in the model group than in the control group (*P* < 0.01), while the protein expression levels were decreased in ATL-III (15, 30, and 60 *μ*mol/L) groups (*P* < 0.05, *P* < 0.01) (Figures 4(a)–4(c)). mRNA levels exhibited a consistent tendency with the changes in protein expression (*P* < 0.01) (Figures 4(d) and 4(e)). The results suggested that the protective effect of ATL-III on H9c2 cells may be related to the inhibition of ERS and downregulation of GRP78 and CHOP.

### 3.5. Effects of ATL-III on PERK, eIF2*α*, and ATF4 Protein and mRNA Expression

Western blot results revealed that the levels of PERK, eIF2*α*, and ATF4 proteins increased in the model group compared with the control group (*P* < 0.01). As compared with the model group, the ATL-III treatment group had a lower expression of PERK, eIF2*α*, and ATF4 (*P* < 0.05; *P* < 0.01) (Figures 5(a)–5(d)). PERK, eIF2*α*, and ATF4 mRNA levels revealed a consistent tendency with changes in protein expression (*P* < 0.01) (Figures 5(e)–5(g)). The findings suggested that the protective effect of ATL-III against ERS in H9c2 cells is related to the downregulation of PERK, eIF2*α*, and ATF4.

### 3.6. Effects of ATL-III on Levels of GRP78, CHOP, and PERK after Using ERS Inhibitor 4-PBA

After inhibiting ERS with 4-PBA, Western blot and RT-qPCR results showed that GRP78, CHOP, and PERK expression levels were elevated in the model group compared to the control group (*P* < 0.01), while they were decreased in ATL-III group, 4-PBA group, and ATL-III+ 4-PBA group (*P* < 0.01). And ATL-III+ 4-PBA group showed the best reduction effect. The data indicated that the inhibition effect of ATL-III on ERS was consistent with that of 4-PBA (Figure 6).

### 3.7. Effects of ATL-III on Levels of PERK, eIF2*α*, and ATF4 after Using PERK Inhibitor GSK2656157

After inhibiting ERS with GSK2656157 (PERK inhibitor), Western blot and RT-qPCR results showed that expression levels of PERK, eIF2*α*, and ATF4 were reduced compared with the control group (*P* < 0.01), while for the inhibition of PERK, its expression of ATL-III group, GSK2656157 group, and ATL-III + GSK2656157 group was reduced compared to the model group (*P* < 0.01), and ATL-III + GSK2656157 group decreased more obviously. The findings indicate that the inhibition effect of ATL-III on the PERK/eIF2*α*/ATF4 pathway was consistent with that of GSK2656157 (Figure 7).

### 3.8. Protective Effect of ATL-III on Apoptosis of H9c2 Cells after Using PERK Inhibitor GSK2656157

We observed cell death after treating cells with GSK2656157 (PERK inhibitor). Flow cytometry results showed that, compared with the model group, the apoptosis rate was significantly lower in ATL-III group (*P* < 0.01), GSK2656157 group, and ATL-III + GSK2656157 group (Figures 8(a) and 8(b)). Western blot results showed that the expression levels of Bax and Caspase-3 were significantly lower in ATL-III, GSK2656157, and ATL-III + GSK2656157 groups compared with the model group (*P* < 0.01), while the expression of Bcl-2 was significantly higher (*P* < 0.01) (Figures 8(c)–8(f)). The findings revealed that ATL-III was consistent with GSK2656157, suggesting a protective effect of ATL-III on H9c2 cells through the PERK pathway.

## 4. Discussion

TCM is widely applied in the prophylaxis and therapy of HF [24]. LGZGD, as one of the widely used TCM, can effectively regulate the cardiac function and structure in HF by ameliorating the microstructural remodeling, reducing the myocardial inflammation injury and myocardial fibrosis [9, 10, 25–27], and can protect myocardial cells by inhibiting apoptosis of H9c2 cells [12]. As one of the active components of LGZGD, previous studies show that ATL-III has a protective effect on myocardial cells [20]. Therefore, in-depth exploration of the protective mechanism of ATL-III against H9c2 cells will be of significant help in the clinical management of HF.

Regulating ERS can improve cardiac function and alleviate CHF process [28]. GRP78 is an important regulator of molecular chaperone and ERS signaling pathway in ER, which reflects the overall level of ERS and is the key to activating ERS signaling pathway [29]. Therefore, in this study, ERS marker GRP78 and key targets of downstream signaling pathway PERK, IRE*α*, and ATF6 were used as molecular docking targets, and molecular docking scores were performed with ATL-III to determine the binding affinity. Molecular docking is a common tool for virtual screening of drugs and their mechanisms of action, which can reveal the interactions between compounds and targets and develop novel drugs [30]. Molecular docking results showed that ATL-III interacted with the ERS key protein GRP78 and PERK, ATF6, and IRE*α*. It is speculated that ATL-III may have potential effects on the inhibition of ERS, which is realized through the PERK pathway. This study further explored whether ATL-III could reduce myocardial cell injury by regulating ERS-mediated apoptosis through subsequent experiments.

ERS is involved in the occurrence and development of various cardiovascular diseases such as hypertension and HF, which is an important target for the management of cardiovascular diseases [31, 32]. ERS is a pathological process due to disruption of ER homeostasis and misfolding of proteins is caused by various factors. In the initial phase of ERS, the UPR is activated. As the main regulator of UPR, GRP78 is activated during cellular stress [33]. GRP78 is a chaperone located in ER, which is widely used as an indicator of inducing ERS [34], and binds to three stress sensors ATF6, IRE1*α*, and PERK to inactivate them under physiological conditions [35]. However, when UPR accumulates, GRP78 dissociates from transmembrane proteins, which are activated by dimerization, triggering downstream pathway protein reactions and initiating ERS signal transduction pathway. Therefore, TM was used in this study to induce ERS injury in H9c2 cells. We found that ATL-III reduced protein and mRNA levels of GRP78 in H9c2 cells, and 4-PBA can prevent protein aggregation and is an effective ERS inhibitor, which can significantly inhibit the expression of GRP78 [36]. The mechanism of ATL-III is consistent with 4-PBA, suggesting that ATL-III attenuates H9c2 cell injury possibly associated with ERS.

PERK is the first to be activated when dissociated from GRP78 [37]. PERK is a serine threonine kinase, which is activated by autophosphorylation and dimerization after disaggregation from GRP78. Activation of PERK leads to phosphorylation of the alpha-subunit of eIF2*α*, leading to attenuation of mRNA translation, protecting cells from the influx of misfolded proteins to cut down protein load in the ER and rebuild the homeostasis of ER. Activation of eIF2*α* inhibited the translation of mRNA, but enhanced the translation and synthesis of ATF4 mRNA, and phosphorylated eIF2*α* can significantly improve the level of ATF4, whose activation requires PERK-dependent eIF2*α* phosphorylation [38]. Phosphorylation-eIF2*α* triggers the synthesis of transcription factor ATF4, which then drives the transcription of the stress protein CHOP and enhances the expression of various protein-encoding genes and protein synthesis levels by binding ATF4. Early in the ERS, the activated PERK signaling pathway can protect cells by inhibiting protein synthesis. However, prolonged ERS triggers apoptosis, not directly, but by activating downstream proapoptotic molecules that push cells toward the death pathway. The expression of CHOP is of great significance in inducing prosurvival to proapoptosis [39]. PERK/eIF2*α*/ATF4 pathway is the leading pathway for activation of CHOP among the three branches of UPR.

CHOP is a crucial factor in ERS-mediated apoptosis by regulating the balance between the Bcl-2 family of pro-apoptotic and anti-apoptotic proteins (Figure 9). Bax is a member of the Bcl-2 family, which consists of the most significant apoptosis regulating factors. Bcl-2 and Bax are antiapoptotic and proapoptotic proteins, respectively, which are the most representative of the Bcl-2 family [40]. CHOP activates the antiapoptotic of Bcl-2 family proteins and mediates transcriptional inhibition [41]. Studies have found that loss of Bax or overexpression of Bcl-2 protects cells from ERS [42]. Therefore, the Bcl-2 family is clearly participating in ERS-induced apoptosis. CHOP downregulates expression of Bcl-2 and increases the translocation of Bax from the cytoplasm to mitochondria, inducing the release of Cyt-c by mitochondria to activate Caspase-3 and induce apoptosis [43]. Apoptosis is important in the development of HF, which is essential to the pathological process of HF [44]. In this study, ATL-III could reduce the levels of phosphorylation-PERK, phosphorylation-eIF2*α*, and ATF4. Further study found the function of PERK in the antiapoptotic process of ATL-III, GSK2656157, and ATL-III + GSK2656157. The findings demonstrated that ATL-III may protect H9c2 cells from ERS damage via the PERK pathway. Subsequently, GSK2656157 was used to further verify the relationship between protective effect of ATL-III on H9c2 cells and the PERK pathway, GSK2656157 is a direct inhibitor of PERK and it turns out that the use of GSK2656157 was consistent with the effect of ATL-III, suggesting that ATL-III protects H9c2 cells through PERK pathway.

## 5. Conclusion

In conclusion, molecular docking was first used to predict ATL-III and potential targets, and the results were verified by in vitro experiments, which were consistent with the prediction. The protection of ATL-III on H9c2 cardiomyocytes may be related to the inhibition of ERS and downregulation of the GRP78/PERK/CHOP signaling pathway, which provided a new target for the management of HF.

## Figures and Tables

**Figure 1:** Docking results of ATL-III with ERS-related molecules of GRP78, IRE*α*, ATF6, and PERK.

**Figure 2:** Effects of ATL-III on H9c2 cell proliferation. (a) Results of H9c2 cells treated with different doses of ATL-III (15, 30, 60, 120, and 240 *μ*mol/L) for 24, 48, and 72 h. (b) Effects of appropriate dose of ATL-III on TM-induced H9c2 cells. Data were mean ± SD; ^*∗∗*^*P* < 0.01 versus control group; ^##^*P* < 0.01 versus model group.

**Figure 3:** Effects of ATL-III on TM-induced apoptosis in H9c2 cells. (a) Flow cytometry assays for the protective effect of ATL-III against apoptosis in H9c2 cells. (b) Apoptosis rate by flow cytometry. (c) Protective effect of ATL-III against apoptosis in H9c2 cells detected by Hoechst/PI double staining. (d) Protein expression levels of Bcl-2 (d, e), Bax (d, f), and Caspase-3 (d, g). Data were mean ± SD; ^*∗∗*^*P* < 0.01 versus control group; ^##^*P* < 0.01 versus model group.

**Figure 4:** Effects of ATL-III on TM-induced GRP78, CHOP protein, and mRNA expression levels. a–c Effects of ATL-III on protein expression levels of GRP78 (a, b) and CHOP (a, c). d-e: effects of ATL-III on mRNA levels of GRP78 (d) and CHOP (e). Data were mean ± SD; ^*∗∗*^*P* < 0.01 versus control group; ^#^*P* < 0.05, ^##^*P* < 0.01 versus model group.

**Figure 5:** Effects of ATL-III on PERK, eIF2*α*, ATF4 protein, and mRNA expression levels caused by TM. a–d: effects of ATL-III on protein expression levels of p-PERK/PERK (a, b), p-eIF2*α*/eIF2*α* (a, c), and ATF4 (a, d). e–g: effects of ATL-III on mRNA levels of PERK (e), eIF2*α* (f), and ATF4 (g). Data were mean ± SD; ^*∗∗*^*P* < 0.01 versus control group; ^##^*P* < 0.01 versus model group.

**Figure 6:** Effects of ATL-III on protein and mRNA expression levels of GRP78, CHOP, and PERK after using ERS inhibitor 4-PBA. a-d: effects of ATL-III on protein expression levels of GRP78 (a, b), CHOP (a, c), and PERK (a, d) after using ERS inhibitor 4-PBA. e-g: effects of ATL-III on mRNA levels of GRP78 (e), CHOP (f), and PERK (g) after using ERS inhibitor 4-PBA. Data were mean ± SD; ^*∗∗*^*P* < 0.01 versus control group; ^#^*P* < 0.05, ^##^*P* < 0.01 versus model group.

**Figure 7:** Influence of ATL-III on PERK/eIF2*α*/ATF4 pathway protein and mRNA expression levels after PERK inhibition by GSK2656157. a-d: effects of ATL-III on protein expression levels of p-PERK/PERK (a, b), p-eIF2*α*/eIF2*α* (a, c), ATF4 (a, d), and CHOP (a, e) after using PERK inhibitor GSK2656157. f-h: effects of ATL-III on mRNA levels of PERK (f), eIF2*α* (g), and ATF4 (h) after using PERK inhibitor GSK2656157. Data were mean ± SD; ^*∗∗*^*P* < 0.01 versus control group; ^#^*P* < 0.05, ^##^*P* < 0.01 versus model group.

**Figure 8:** Effects of ATL-III on apoptosis after inhibition of PERK. (a) Protective effect of ATL-III on apoptosis after using PERK inhibitor GSK2656157 was detected by flow cytometry. (b) Apoptosis rate by flow cytometry after treatment with the PERK inhibitor GSK2656157. c-f: protein expression levels of Bcl-2 (c, d), Bax (c, e), and Caspase-3 (c, f) after treatment with the PERK inhibitor GSK2656157. Data were mean ± SD; ^*∗∗*^*P* < 0.01 versus control group; ^#^*P* < 0.05, ^##^*P* < 0.01 versus model group.

**Figure 9:** Mechanism of ATL-III acting on the GRP78/PERK/CHOP signaling pathway.

**Table 1:** Primers used in RT-qPCR.

Primers		Sequence 5′ to 3′
GRP78	Forward	CGGAGGAGGAGGACAAGAAGGAG
	Reverse	ATACGACGGTGTGATGCGGTTG

CHOP	Forward	CTAGGAAACGGAAACAGAGTGGTCAG
	Reverse	TCCTCTCATTCTCCTGCTCCTTCTC

PERK	Forward	TGGGATGTCGCCGATGGGATAG
	Reverse	AATTCCACTTCTCACTGCCGCTTC

eIF2*α*	Forward	GCGAATTGTGGCAGGTTTCTTGG
	Reverse	TAGGCTCCTCACTAGGCACTTCAC

ATF4	Forward	AGTCTGCCTTCTCCAGGTGTTCC
	Reverse	GCTGCTGTCTTGTTTTGCTCCATC

*β*-actin	Forward	CCCATCTATGAGGGTTACGC
	Reverse	TTTAATGTCACGCACGATTTC

**Table 2:** Docking of native ligand with GRP78, PERK, IRE*α*, and ATF6.

Targets	Vina score
GRP78	−7.5
PERK	−8.1
IRE*α*	−7.9
ATF6	−6.4

## Data Availability

The data used during the study are available from the corresponding author upon request.
